The article "RUNX3-Regulated GALNT6 Promotes the Migration and Invasion of Hepatocellular Carcinoma Cells by Mediating O-Glycosylation of MUC1" was retracted in 2023. Reasons: signs of a paper mill; suspected computer-generated content; unreliable results or conclusions; concerns about the data.

# RUNX3-Regulated GALNT6 Promotes the Migration and Invasion of Hepatocellular Carcinoma Cells by Mediating O-Glycosylation of MUC1

**DOI:** 10.1155/2022/2959846

**Published:** 2022-07-21

**Authors:** Fei Gao, Gang Zheng

**Affiliations:** Department of Biliary-Pancreatic Surgery, Shanxi Bethune Hospital, Shanxi Academy of Medical Sciences, Tongji Shanxi Hospital, Third Hospital of Shanxi Medical University, China

## Abstract

**Background:**

Hepatocellular carcinoma (HCC) is a leading cause of cancer-related death worldwide. Dysregulation of messenger RNAs (mRNA) has been recognized to be associated with HCC carcinogenesis and development. Polypeptide GalNAc Transferase 6 (GALNT6), an O-type glycosyltransferase, has been confirmed as tumor promoter in different cancers. However, the function of GALNT6 in HCC remains to be studied.

**Methods:**

RT-qPCR and western blot experiments were, respectively, performed for evaluating RNA expressions and protein levels. Supported by bioinformatics analysis, mechanism assays were conducted for validating the potential relation between different genes. Functional assays were implemented to analyze HCC cell migration and invasion after different transfections.

**Results:**

GALNT6 was aberrantly upregulated in HCC cells. Knockdown of GALNT6 could repress HCC cell migration and invasion. RUNX3 was verified to bind to GALNT6 promoter and activate GALNT6 transcription. GALNT6 depletion led to inhibited O-glycosylation and aggravated degradation of MUC1. MUC1 overexpression could rescue the impeded HCC cell migration and invasion induced by GALNT6 knockdown.

**Conclusion:**

To sum up, GALNT6 transcriptionally activated by RUNX3 mediated the O-glycosylation of MUC1, thus exerting promoting influence on HCC cell migration and invasion.

## 1. Introduction

Hepatocellular carcinoma (HCC), the most common type of primary liver cancer, severely affects human life worldwide for its high morbidity and mortality [1]. Undoubtedly, nondrug therapies and drug regimens for HCC treatment have been improved in recent years. Specifically, hepatic resection and liver transplantation are favorable to early and mid-stage HCC patients, and medications including sorafenib, lenvatinib, and nivolumab can be applied to treat patients with advanced HCC [2, 3]. However, an increase in HCC morbidity has been observed in past decades [4], and the increasingly elevated financial stress is still a chief reason of delayed treatment [5]. Additionally, patients diagnosed with HCC still suffer from poor prognosis and frequent recurrence [6]. Therefore, it is essential to understand the inner molecular mechanisms associated with HCC carcinogenesis and progression, thus contributing to development of new strategies for HCC diagnosis and treatment.

Glycosylation is considered a primary posttranslational modification of proteins, and the previous literature has unveiled the integral link between glycosylation changes and the progression of some malignancies [7, 8]. Abnormal O-glycosylation has been suggested as an effector in modulating various cellular activities, tumor growth, and metastasis [9, 10]. The N-acetylgalactosaminyltransferases (GalNac-Ts; GALNTs) are a family of enzymes that catalyze O-glycosylation of various molecules, and GALNT-mediated O-glycosylation has been reported to influence protein processing that is significantly associated with pathophysiological processes [11, 12]. GALNT14, aberrantly upregulated in various malignancies, has been suggested as a putative marker for prediction of therapeutic outcomes in some cancers, including HCC [13]. As a member of this family, GALNT6 has been reported as a facilitator for tumor metastasis and progression [14]. More specifically, GALNT6 can contribute to invasion and epithelial-mesenchymal transition (EMT) of lung adenocarcinoma cells, which is essential to tumor metastasis, via the mediation on chaperone protein GRP78 O-glycosylation [15]. GALNT6 has also been validated to accelerate breast cancer metastasis via the modulation on *α*2M O-glycosylation and PI3K/Akt signaling activation [12]. However, the specific molecular mechanisms of GALNT6 in HCC metastasis and development remain to be elucidated.

The aim of this study was to investigate the influences of GALNT6 on migration and invasion of HCC cells, with O-glycosylation taken into consideration, thus offering a novel insight for understanding HCC.

## 2. Material and Methods

### 2.1. Cell Culture

Normal liver cell line (THLE-2) and three HCC cell lines (HuH-7, Hep 3B, and Li-7) were all purchased from American Type Culture Collection (ATCC; Manassas, VA, USA). HuH-7 and Hep 3B cells were, respectively, cultured in Dulbecco's modified Eagle's media (DMEM; low glucose) containing 10% fetal bovine serum (FBS) and Eagle's Minimum Essential Medium (EMEM) containing 10% FBS. Li-7 cells were cultivated in RPMI1640 medium supplemented with 10% FBS. BEGM medium with additional 70 ng/mL phosphoethanolamine, 5 ng/mL epidermal growth factor (EGF), and 10% FBS was used to culture THLE-2 cells. Human embryonic kidney 293T cells were provided by China National Institutes for Food and Drug Control and cultivated in DMEM medium containing 10% FBS and antibiotics. All cells were cultured in a humidified atmosphere with 5% CO_2_ at 37°C.

### 2.2. Cell Transfection

Small interfering RNAs (siRNAs) including si-GALNT6-1/2/3, si-RUNX3-1/2/3, si-EBF1-1/2/3, and si-CTCF-1/2/3 were generated to knockdown corresponding genes in HCC cells. The whole sequence of RUNX3 or MUC1 was subcloned into pcDNA3.1 vectors for overexpression of RUNX3 or MUC1 in HCC cells. Scramble siRNAs or empty vector pcDNA3.1 was acquired as negative controls. Plasmid transfection was completed with application of Lipofectamine 2000 in strict accordance with user protocol.

### 2.3. Reverse Transcription Quantitative Real-Time Polymerase Chain Reaction (RT-qPCR)

After isolation of total RNA from cells with TRIzol reagent, the extracted RNA was reversely transcribed into cDNAs with Reverse Transcriptase Kit. RNA expression analysis was conducted using qRT-PCR kit. The expression of the detected gene was measured by the 2^-*ΔΔ*CT^ method. *β*-Actin served as endogenous control.

### 2.4. Transwell Migration and Invasion Assay

After transfection of indicated plasmids for 24 h, the cells were added into the apical transwell chamber containing serum-free medium with (for invasion) or without (for migration) Matrigel. The basal Transwell chamber was added with 10% FBS. After 24 h, the cells in the inside of the chambers were wiped off and the successfully migrated or invaded cells on the outside of the chambers were fixed with methanol and dyed with crystal violet. Cell number in 5 randomly selected fields was counted under a microscope.

### 2.5. Wound Healing Assay

Transfected cells were planted into a 6-well plate and cultured in a DMEM overnight. After scratches were made with a plastic tip, cells were continuously cultured in serum-free DMEM. Wound closure was viewed at 0 h and 24 h, respectively.

### 2.6. DNA Pull down Assay

For DNA pull down, the biotin-labeled GALNT6 promoter and negative control probes were conjugated with beads for coculturing with the protein extracts from HCC cells for 2 h. Proteins were purified and subjected to western blot analysis.

### 2.7. Western Blot

After the cells were lysed in RIPA buffer, PROTTOT-1KT and Bradford Protein Assay Kit were, respectively, applied to extract total protein and to detect the concentration of the proteins in cell lysates. Later, the proteins treated with 10% SDS-PAGE were transferred onto the PVDF membranes, which were blocked with 5% skimmed milk and then cocultivated with specific primary antibodies against RUNX3, *β*-actin, MUC4, or MUC1 overnight at 4°C. Subsequently, secondary antibodies were added for further cultivation at room temperature. Enhanced chemiluminescence (ECL) detection system was applied to visualize immunoreactive bands.

### 2.8. Luciferase Reporter Assay

293T cells were cultured in a 24-well plate and grown up to 70% coverage. The pGL3 Luciferase Reporter Vectors containing GALNT6 promoter with the wild-type or mutant binding site of RUNX3 were constructed. The constructed vectors, as well as pcDNA3.1-RUNX3 or negative control (pcDNA3.1), were transfected into 293 T cells, respectively. The luciferase assay was performed according to the manufacturer's protocol.

### 2.9. Chromatin Immunoprecipitation (ChIP)

ChIP RNA-Binding Protein Immunoprecipitation Kit was applied in ChIP assay for the investigation into the putative correlation between RUNX3 and GALNT6 promoter. The crosslinked chromatin was first cut into fragments (200-1000 bp) for immunoprecipitation with primary antibody against IgG or RUNX3, together with magnetic beads. Subsequent to elution and purification, the precipitated DNAs were analyzed via RT-qPCR.

### 2.10. Coimmunoprecipitation (Co-IP)

The cells were lysed by cold lysis buffer containing complete protease inhibitors and centrifuged at 14,000 × g for 20 min at 4°C. The supernatant from cell lysates was incubated with antibody against IgG or GALNT6. The immunocomplexes were then associated with Protein A-Sepharose. The proteins were then subjected to analysis through western blot.

### 2.11. Statistical Analysis

SPSS 22.0 software was used for the statistical analyses in present study. Each experiment was performed for at least three times. All data were demonstrated as the mean ± standard derivation (SD). Student's *t*-test was applied for the comparison of two groups, while ANOVA was applied to examine the differences of three or more groups. Data was considered to indicate statistical significance with two-sided *P* < 0.05.

## 3. Results

### 3.1. GALNT6 Facilitates Migration and Invasion of HCC Cells

Previous studies have unveiled the oncogenic role of GALNT6 in different cancers, including breast cancer and lung adenocarcinoma [12, 15]. Hence, we aimed to explore the putative role of GALNT6 in HCC. Based on UALCAN (http://ualcan.path.uab.edu/index.html), GALNT6 was discovered to be aberrantly upregulated in HCC tissues (Figure 1(a)). RT-qPCR analysis was then done for the measurement of GALNT6 expression in different cell lines, and the results of which showed GALNT6 expression was much higher in HCC cells than in THLE-2 (Figure 1(b)). Furthermore, Li-7 and Hep 3B (with the highest GALNT6 expression) were selected for subsequent functional assays. The knockdown efficiency of si-GALNT6 was determined in advance (Figure S1A), and si-GALNT6-1/2 was chosen for the higher efficiency. It was suggested in RT-qPCR analysis that GALNT6 depletion led to a decrease in the levels of MMP2 and MMP9 (invasion-related genes), suggesting the suppressive impacts of GALNT6 knockdown on HCC cell invasion (Figure 1(c)). Wound healing outcomes indicated that the migratory ability of HCC cells could be overtly weakened by GALNT6 silence (Figure 1(d)). The inhibitory influences of GALNT6 knockdown on cell migration and invasion in HCC were further confirmed by Transwell experiments as a decline in migrated and invaded cells could be observed as a result of si-GALNT6-1/2 transfection (Figures 1(e) and 1(f)). The above findings together prove that GALNT6, upregulated in HCC tissues and cell lines, can contribute to cell migration and invasion in HCC.

### 3.2. RUNX3 Is the Transcriptional Activator of GALNT6

Next, our emphasis was laid on exploration into the molecular mechanism contributing to the aberrantly high expression of GALNT6 in HCC. It was learnt from previous research that transcriptional factors might activate the transcription of the target genes via binding to the corresponding promoters [16]. Thus, UCSC (http://genome.ucsc.edu/) was applied to predict transcription factors of GALNT6, and three genes (RUNX3, EBF1, and CTCF) were picked out as the candidate transcription factors for their highest cluster score (Figure 2(a)). After determining the respective knockdown efficiency of si-RUNX3, si-CTCF, and si-EBF1 (Figure S1B-D), it was manifested in RT-qPCR results that only RUNX3 depletion resulted in an overt reduction in GALNT6 expression (Figure 2(b)). The binding site of RUNX3 and GALNT6 was predicted on JASPAR (https://jaspar.genereg.net/), and the predicted sequence with the highest score was GGAACCACAACA (Figure 2(c)). In DNA pull down assay, RUNX3 was discovered to be abundantly pulled down by Bio-GALNT6 promoter WT, suggesting the affinity between RUNX3 and GALNT6 (Figure 2(d)). Moreover, according to outcomes of luciferase reporter assay, RUNX3 overexpression could obviously elevate the luciferase activity of pGL3-GALNT6 promoter WT, while that of pGL3-GALNT6 promoter MUT was hardly altered under the same condition, which reflected that RUNX3 could activate the transcription of GALNT6 (Figure 2(e)). The binding correlation between RUNX3 and GALNT6 promoter was further confirmed by ChIP assay (Figure 2(f)). To conclude, RUNX3 can transcriptionally modulate GALNT6 in HCC cells.

### 3.3. GALNT6 Mediates O-Glycosylation T of MUC1

Based on recent studies, the oncogenic role of GALNT6 in breast cancer and lung adenocarcinoma is dependent on O-glycosylation [12, 15]. Therefore, we also tended to explore whether GALNT6 modulation mechanism in HCC cells was associated with O-glycosylation of its downstream protein. We firstly searched on STRING (https://string-db.org/) to predict the interacting proteins of GALNT6 and applied UALCAN to predict the expression patterns of the top four proteins with highest score (Figure 3(a)). The expression of MUC5AC in LIHC could not be obtained from UALCAN. Among the other three candidates, MUC1 and MUC4, upregulated in LIHC tissues, were chosen. The results of Co-IP assay revealed the stronger binding between MUC1 and GALNT6 than that between MUC4 and GALNT6, so MUC1 was determined as our research target (Figure 3(b)). Then, several O-glycosylation sites in MUC1 were observed based on NetOGlyc-4.0 (https://services.healthtech.dtu.dk/service.php?NetOGlyc-4.0) prediction (Figure 3(c)). As illustrated in Figure 3(d), GALNT6 depletion resulted in a decline in MUC1 protein level pulled down by vicia villosa agglutinin (VVA), mirroring that GALNT6 might mediate MUC1 O-glycosylation. For further confirmation, Li-7 cells were treated with O-glycosylation inhibitor Benzyl-alpha-GalNAc (BAG). According to VVA lection pull down and western blot analysis, GALNT6 overexpression could contribute to MUC1 O-glycosylation (Figure 3(e)). Additionally, HCC cells transfected with si-NC or si-GALNT6-1 were subjected to cycloheximide (CHX) treatment and the results of western blot analysis verified that GALNT6 depletion could accelerate MUC1 protein degradation (Figure 3(f)). Taken together, GALNT6 mediates O-glycosylation of MUC1 in HCC cells.

### 3.4. GALNT6 Influences HCC Cell Migration and Invasion via Modulation on MUC1

The validity of GALNT6/MUC1 regulatory axis in HCC cells was next investigated by performing rescue experiments. MUC1 overexpression efficiency was firstly detected via RT-qPCR (Figure S1E). Similarly, RT-qPCR analysis was done to examine changes in MMP2 and MMP9. Reduction in MMP2 and MMP9 levels, resulting from GALNT6 silence, was discovered to be recovered by MUC1 overexpression (Figure 4(a)). Supported by wound healing assay, it was discovered that MUC1 overexpression could reverse the inhibition on cell migration which was attributed to GALNT6 silence (Figure 4(b)). The outcomes of Transwell assays further confirmed that the suppressive influences of GALNT6 depletion on cell migration and invasion could be completely countervailed by MUC1 overexpression (Figures 4(c) and 4(d)). To sum up, GALNT6/MUC1 axis is a crucial modulator for HCC cell migration and invasion.

## 4. Discussion

HCC accounts for more than 90% of total hepatic carcinoma cases [17]. As one of the most prevailing malignancies around the world, HCC incidence is still increasing [18]. Normally, infection of chronic hepatitis B and hepatitis C exists as the major reason for HCC induction, while addiction to alcohol, dietary exposure to aflatoxins or aristolochic acid, and liver disease metastasis are all risk factors of HCC [19, 20]. Advancement in molecular pathology has brought about improvement in HCC diagnosis, detailed subtype classification, and prognosis prediction, which also provides help for application of treatment [21].

RNAs, either coding RNAs or noncoding RNAs, are recognized as important effectors in the tumor initiation, progression, and metastasis [22]. GALNT6, encoding a number of the GalNAc-T family of enzymes [23], has been discovered as tumor promoters in various diseases [14, 24]. Consistently, after we confirmed that GALNT6 was upregulated in HCC tissues and cell lines, we also verified GALNT6 could promote HCC cell migration and invasion, implying GALNT6 was an oncogene in HCC.

To probe into the underlying mechanism contributing to the upregulation of GALNT6 in HCC cells, we conducted bioinformatics analysis and mechanism assays to ravel out the transcription factor of GALNT6. As a result, RUNX3 was discovered as the transcription factor promoting the transcription of GALNT6. Subsequently, considering the role of GALNT6 as an O-type glycosyltransferase [25], we aimed to figure out the downstream protein whose O-glycosylation could be mediated by GALNT6. With utilization of STRING and UALCAN databases, as well as Co-IP verification, MUC1, an interacting protein of GALNT6 with aberrantly high expression in HCC was screened out. MUC1 has been much investigated regarding to cancer development. For instance, MUC1 as a ceRNA participant has been discovered to promote ovarian cancer progression [26]. The O-glycans of MUC1 has also been reported as a crucial effector in tumor development [27]. As MUC1 is a transmembrane mucin glycoprotein expressed on the surface of almost all epithelial cells, vaccine based on MUC1 has been regarded as a promising method for cancer treatment [28]. In our study, implementation of VVA pull down assay and western blot assay jointly certified MUC1 O-glycosylation mediated by GALNT6 could lessen the degradation of MUC1 protein in HCC cells. The rescue assays further corroborated that GALNT6 exacerbated HCC cell migration and invasion via positively regulating MUC1 expression.

There are still some limitations in this study included. Xenograft models were not involved to analyze the influence of RUNX3/GALNT6/MUC1 axis on HCC progression in vivo, and clinical samples were not obtained for certifying the correlation between GALNT6 expression and pathological features. Nevertheless, this study could still provide a novel perspective for understanding the molecular regulatory mechanism implicated in HCC.

Collectively, our study indicated GALNT6 was overexpressed in HCC. GALNT6 transcriptionally upregulated by RUNX3 could mediate the O-glycosylation of MUC1, thus positively regulating MUC1 expression to ameliorate HCC cell migration and invasion.

## Figures and Tables

**Figure 1:** GALNT6 is high expressed in HCC and promotes HCC cell migration and invasion. (a) UALCAN predicted the expression pattern of GALNT6 in HCC tissues and normal tissues. (b) GALNT6 level in different cell lines was analyzed via RT-qPCR. (c) Invasion-related genes (MMP2 and MMP9) were quantified through RT-qPCR after cells were transfected with si-NC or si-GALNT6. (d) The migratory ability of HCC cells was analyzed with application of wound healing assay. (e, f) Transwell assays were carried out for validating HCC cell migratory and invasive capabilities before and after GALNT6 silence. ^∗^*P* < 0.05, ^∗∗^*P* < 0.01.

**Figure 2:** GALNT6 is transcriptionally activated by RUNX3 in HCC cells. (a) UCSC was applied to predict the transcription factors of GALNT6. (b) The expression variation of GALNT6 before and after knockdown of RUNX3, CTCF, or EBF1 was analyzed through RT-qPCR. (c) JASPAR was utilized to predict the binding sites of RUNX3 and GALNT6 promoter. (d) Wild-type or mutated GALNT6 promoter was biotinylated to pull down RUNX3 and the result was analyzed via western blot. (e) Luciferase activity of pGL3-GALNT6 promoter WT/MUT was measured in HCC cells with pcDNA3.1 or pcDNA3.1-RUNX3 transfected. (f) RIP assay validated the cohesion between RUNX3 and wild-type or mutated GALNT6 promoter in HCC cells. ^∗∗^*P* < 0.05.

**Figure 3:** O-glycosylation of MUC1 is mediated by GALNT6. (a) STRING was utilized for predicting the interacting proteins of GALNT6 while UALCAN was applied to obtain the expression patterns of the candidates. (b) Co-IP assay was performed to prove the interaction between GALNT6 and candidate proteins. (c) The O-glycosylation sites of MUC1 were predicted with the help of NetOGlyc-4.0 database. (d) Lectin pull down with VVA and western blot assay were applied to analyze influence of GALNT6 knockdown on MUC1 O-glycosylation. (e) MUC1 O-glycosylation under indicated condition (BAG treatment or GALNT6 upregulation) was analyzed with application of VVA. (f) CHX was used to inhibit protein synthesis in Li-7 and Hep 3B cells with or without GALNT6 depletion and MUC1 level was measured through western blot.

**Figure 4:** GALNT6 affects HCC migration and invasion by positively modulating MUC1 expression. (a) MMP2 and MMP9 levels were quantified through RT-qPCR in HCC cells with different transfections, including si-NC, si-GALNT6-1, si-GALNT6-1+pcDNA3.1, and si-GALNT6-1+pcDNA3.1-MUC1. (b) The wound healing width at different time points was measured and analyzed to reflect the migratory ability of HCC cells in different groups. (c) HCC cell migration and invasion was examined through Transwell assays. ^∗∗^*P* < 0.01.

## Data Availability

Data will be available upon reasonable request.

## Supplementary Materials

Supplementary Materials Figure S1: (A) GALNT6 was knocked down in Li-7 and Hep 3B cell lines with transfection of si-GALNT6-1/2/3. (B–D) RUNX3, CTCF, or EBF1 was, respectively, silenced in HCC cells and the knockdown efficiency was proved through RT-qPCR. (E) MUC1 overexpression was accomplished by transfecting of pcDNA3.1-MUC1. ^∗∗^*P* < 0.01.
